RETRACTED

# Overexpression of Rad51 Predicts Poor Prognosis in Colorectal Cancer: Our Experience with 54 Patients

**DOI:** 10.1371/journal.pone.0167868

**Published:** 2017-01-18

**Authors:** Yan Li, Wei-ya Wang, Jiang-hong Xiao, Feng Xu, Dian-ying Liao, Li Xie, Jin Wang, Feng Luo

**Affiliations:** 1 Department of Radiation Oncology, Cancer Center, West China Hospital, Sichuan University, Chengdu, China; 2 Department of Pathology, West China Hospital, Sichuan University, Chengdu, China; 3 Center for Radiation Physics and Technology, Cancer Center, West China Hospital, Sichuan University, Chengdu, China; 4 Lung Cancer Center, West China Hospital, Sichuan University, Chengdu, China; State University of New York, UNITED STATES

## Abstract

**Background:**

Aberrant Rad51 expression is implicated in the progression of human malignancies. However, the role of Rad51 in colorectal cancer (CRC) remains undefined. This study aimed to establish a relationship between Rad51 and clinicopathologic features of CRC.

**Methods:**

We retrospectively examined the paraffin-embedded tissue samples obtained from 54 patients with CRC who had received surgical therapies at our institution during 2006–2008. Rad51 expression in adenocarcinoma, paracancerous tissue, and normal colonic tissue was determined by immunohistochemistry. The correlation between Rad51 immunoreactivity and clinicopathologic features of these patients was evaluated.

**Results:**

Rad51 immunoreactivity was detected in 67% of adenocarcinoma, 48% of paracancerous tissue, and 27% of normal colonic mucosa. Rad51 expression in adenocarcinoma was significantly higher than normal colonic tissue (*p* < 0.05). Rad51 was also overexpressed in poorly differentiated tumors and tumor samples from patients with lymph node metastasis (*p* < 0.05). Patients with Rad51 overexpression had a 69% two-year survival, 49% three-year survival, and 16% five-year survival, considerably worse than patients with negative Rad51 expression (*p* < 0.05).

**Conclusion:**

Our data suggest that Rad51 overexpression is correlated with malignant phenotypes of CRC and may predict poor prognosis for these patients.

## Introduction

Colorectal cancer (CRC) is a third frequently diagnosed human malignancy with a mortality rate greater than 33%, and each year there are over one million new CRC cases reported worldwide [1]. Currently, available regimens for CRC include surgery, radiotherapy, and chemotherapy, and the combination of these regimens has slightly improved the overall survival. CRC patients carrying the KRAS mutation may have an additional option for the therapy targeting the EGFR signaling pathway [2, 3]. Despite these advances, local recurrence, distant metastasis and eventual relapse remain common with many CRC patients who have received all these treatments. Hence, it is clinically desirable to explore novel diagnostic markers and pathways that may be targeted for developing new CRC therapies.

RETRACTED

DNA repair pathway has been considered a promising target for cancer therapy development, as the chromosomal integrity is a prerequisite for normal cell division. Homologous recombination involves chromosomal pairing and exchange of the DNA strands, the process catalyzed by the nuclear protein Rad51 [4, 5]Rad51 has lately received much attention for its implication in tumor progression. There is evidence for the association of abnormal Rad51 expression with tumor resistance to chemotherapy [6]. For example, small cell lung cancer cells with Rad51 overexpression showed enhanced tolerance to anticancer drug etoposide VP-16 [7]. On the other hand, tumor cells in which Rad51 expression was suppressed by RNA interference became susceptible to chemotherapeutic drugs [8]. Likewise, treatment with cisplatin and nitrogen mustard induced Rad51 expression in ovarian and testicular cancer cells along with an increase in their resistance to chemotherapy [9]. Furthermore, suppression of Rad51 expression through RNA interference directly enhanced the sensitivity of tumor cells to a cisplatin-based chemotherapy [10].

Aberrant Rad51 expression also has a profound impact on tumor response to radiotherapy, which generates extensive double-strand breaks and promotes tumor cell apoptosis. In the presence of overexpressed Rad51, tumor cells often show a greater resistance to the radiation-mediated apoptosis, whereas tumor cells with downregulated Rad51, through either genetic changes or immunological inhibitions, show hypersensitive to radiation [6]. For example, antisense oligonucleotide-mediated inhibition of Rad51 expression in rat M5S skin cancer cells or rat 203G glioma cells resulted in a significant decrease in tumor cell proliferation along with an increased susceptibility to radiation [11]. Similarly, inhibition of Rad51 by antisense oligonucleotides in LNCaP prostate cancer cells has also resulted in a substantial increase in their response to radiation [12].

Expression of Rad51 is subjective to the regulation by tyrosine kinases and attenuated upon treatment with tyrosine kinase inhibitors such as Gleevec [13]. Tumor cells treated with Gleevec showed considerably less nuclear Rad51 foci in the irradiated cells compared to the untreated cells [14]. Overexpression of Rad51 has also been associated with carcinomas originating from breast, pancreas, head and neck, lung, and esophagus, and often correlated with poor prognosis of those patients [15–20]. Yet, there are few reports in CRC. The presented study was designed to evaluate the clinicopathologic correlation of Rad51 expression with CRC progression and prognosis through a retrospective examination of 54 CRC patients diagnosed and treated at our hospital during 2006–2008.

RETRACTED

## Materials and Methods

### Specimens

Paraffin-embedded specimens were prepared with tissue samples collected from 54 patients who had been diagnosed with colorectal adenocarcinoma at the stages of T_1-4_N_0-2_M_0_ and received radical surgeries followed by chemotherapies and/or radiotherapies during the period of January 2006 to December 2008 at the West China Hospital of Sichuan University. All participants have provided the written consent. The study and consent procedure were approved by the Institutional Ethics Committee at Sichuan University. All tumors were conventional colonic adenocarcinoma. In addition to tumors, paracancerous and normal colonic tissues were also collected. The specimens were fixed in 10% formaldehyde and paraffin-embedded on a routine basis with conventional methods.

### Immunohistochemistry

The archived paraffin blocks were cut into 4 μm sections and incubated at 56°C overnight. After deparaffinization, the sections were treated with 3% hydrogen peroxide to inactivate endogenous peroxidase, and antigen retrieved in citrate. The sections were placed in PBS containing 5% normal goat serum and incubated at 37°C. After 30 min, the sections were incubated with either rabbit anti-human Rad51 antibody (Chemicon, Shanghai, China) at 1:300 dilution or PBS alone as a control. After rinsing three times with PBS, the samples were added with biotinylated goat anti-rabbit polyclonal antibody (Zhong Shan Golden Bridge Biotechnology Co. Beijing, China) and incubated at 37°C for 40 min followed by rinsing three times with PBS. The treated sections were further incubated with the antibody against streptavidin peroxidase (Zhong Shan Golden Bridge Biotechnology Co. Beijing, China) at 1: 200 at 37°C for 30 min. Finally, the sections were stained with DAB (Zhong Shan Golden Bridge Biotechnology Co. Beijing, China). The same sections were further stained for 4 min with hematoxylin followed by rinsing with distilled water, destained with acid alcohol, and stained with eosin. The sections were dehydrated in ethanol for 3 min, cleared with xylene, dried and covered with mounting medium (Zhong Shan Golden Bridge Biotechnology Co. Beijing, China) [21].

### Staining scores

The slides were examined under a light microscope at 200X magnification. The positively stained cells within five microscopic fields corresponding to diseased areas were counted and normalized with the formula: the percentage of positive cells = (number of positive cells / number of total cells) × 100%. Rad51 immunopositivity was mainly present in the nuclei and manifested in varying colors from brown to light yellow. A semi-quantitative counting method was used to score Rad51 expression based on both staining intensity and percentage of positive cells. The staining intensity, as compared to the background, was scored as follows: 0 = no staining; 1 = light yellow; 2 = brownish yellow; and 3 = brown. The percentage of positive cells was scored as follows: 1 = 6% -25% of cells stained positive; 2 = 26% -50%; 3 = 51% -75%; and 4 = greater than 76%. We defined a sample positive for Rad51 expression when the sample had a combined score for staining intensity and percentage of positive cells greater or equals to 3, and a sample negative if the combined score was less than 3.

RETRACTED

### Statistical methods

All data were analyzed with SPSS 16.0 (IBM Corporation, Armonk, New York, USA). Uni-variate analysis was used to analyze the correlation of Rad51 expression with different clinical characteristics. Kaplan-Meier survival analysis was used to analyze the relationship between Rad51 expression and patient survival. P < 0.05 was considered statistically significant.

## Results

### Rad51 expression in CRC, paracancerous and normal colonic tissues

We first determined the Rad51 expression in colorectal tissues by immunohistochemistry. Positively stained cells displayed yellow, buffy and brown granules in the nuclei. As summarized in Table 1, tumor samples had an overall staining intensity score of 3, whereas paracancerous and normal colonic tissue samples had 2. The percentage of positive cells was 67% in tumor samples, 48% in paracancerous tissue, and 27% in normal colonic tissue. Overall, Rad51 expression in adenocarcinoma was statistically higher than in the normal colonic tissue (p < 0.001), but was not significantly different compared to the paracancerous tissue (Fig 1) (p > 0.05). Also, no significant difference in Rad51 expression was found between the paracancerous and normal tissues (p > 0.05).

**Table 1:** Expression of Rad51 in three groups.

Group	n	Staining intensity score	Rad51 expression	Rad51 positive score	p-value
**Adenocarcinoma**	54	3	67%	6.12 ± 1.22	p < 0.001
**Paracancerous tissue**	54	2	48%	3.26 ± 0.98	
**Normal colonic tissue**	54	2	27%	3.21 ± 1.01	

**Fig 1:** Rad51 expression in adenocarcinoma, paracancerous and normal colonic tissue. Rad51 expression in adenocarcinoma was statistically higher than in the normal colonic tissue. * p < 0.001.

### Rad51 overexpression is associated with the poor differentiation and lymph node metastasis

We further noted Rad51 expression was higher in poorly differentiated tumors than in tumors with a well differentiated histology (Fig 2 and Table 2), and higher in patients with lymph node metastasis than in those with negative lymph nodes (Fig 3 and Table 2) (p < 0.05). However, there was no significant correlation between Rad51 expression with patient's gender, age, tumor size or T stage (p > 0.05).

RETRACTED

**Fig 2:** Immunohistochemical analysis of Rad51 expression in CRC tissues. (**A)** Rad51 was overexpressed in a poorly differentiated CRC. Cells with positive Rad51 expression showed yellow, buffy and brown granules in the nuclei. (**B)** Rad51 staining was negative in a well differentiated CRC. (**C)** H&E staining of a poorly differentiated CRC. (**D)** H&E staining of a well differentiated CRC. Representative images with original magnification at 200X. **(E)** Quantitation of Rad51 expression in poorly differentiated versus well differentiated tumors. * p = 0.006.

**Fig 3:** Rad51 expression is associated with lymph node metastasis. Strong Rad51 immunoreactivity was detected in a tumor with lymph node metastasis (**A**), but not in a tumor with negative lymph node metastasis (**B**). Corresponding H&E staining of a metastatic lymph node (**C**) and a negative lymph node (**D**). Representative images with original magnification at 200X. **(E)** Quantitation of Rad51 expression in patients with lymph node metastasis versus patients without. * p = 0.002.

**Table 2:** Correlation of Rad51 expression with clinicopathological characteristics.

Characteristics	n	Staining intensity score	Rad51 expression	Rad51 positive score (*χ*_2_)	p-value
**Sex**					
**Male**	34	3	69%	0.635	0.425
**Female**	20	3	62%		
**Age**					
**>= 60 years**	38	3	67%	0.044	0.083
**< 60 years**	16	3	51%		
**Tumor size**					
**>= 5 cm**	42	3	58%	0.482	0.487
**< 5 cm**	12	3	54%		
**Tumor differentiation**					
**Well differentiated**	22	3	37%	7.517	0.006
**Poorly differentiated**	32	3	78%		
**T stage**					
**T1 and T2**	15	3	61%	0.110	0.74
**T3 and T4**	39	3	68%		
**N stage**					
**N-**	15	3	29%	12.047	0.002
**N+**	39	3	75%		

### Rad51 overexpression predicts poor prognosis in CRC

Finally, we found Rad51 expression was significantly correlated with poor prognosis, as indicated by the Kaplan-Meier analysis (Fig 4). Patients with Rad51 overexpression had a 69% two-year survival, 49% three-year survival, and 16% five-year survival. In contrast, patients with negative Rad51 expression had better clinical outcomes (p < 0.05) with a 90%, 82%, and 78% two-year, three-year and five-year survival, respectively.

**Fig 4:** Kaplan-Meier survival analysis of CRC patients with or without Rad51 overexpression. The survival rate for patients with Rad51 overexpression was significantly lower than those without Rad51 amplification.

RETRACTED

## Discussion

One recent effort to increase the efficacy of chemotherapy and/or radiotherapy has been focused on the inhibition of DNA repairing. DNA repairing requires the action of Rad51, which allows tumor survival and shields tumor cells from DNA damages induced by therapies. Overexpression of Rad51 in tumor cells may also cause excessive homologous recombination and exchanges between the sister chromatids, leading to genetic instability [22]. In this study, we showed that Rad51 expression was elevated in CRC in our cohort of 54 patients, and was significantly higher compared to the normal colonic tissue. This finding is in line with the notion that Rad51 overexpression is implicated in the progression of CRC. Interestingly, we did not observe a significant difference between carcinoma and paracancerous tissue, which could be explained by the infiltration of tumorous cells into the areas immediately adjacent to the lesions.

Rad51 overexpression has been observed in various tumor cell lines, including the cervical cancer Hela cells and MCF-7 breast cancer cells, compared to the cells derived from non-cancerous tissues [23]. Enhanced Rad51 expression was also found in 5%-30% of the pancreatic cancer cell lines and in over 66% of primary pancreatic cancer specimens [22]. A recent microarray analysis also revealed an 11-fold increase of Rad51 mRNA in pancreatic carcinoma compared to the control samples [24]. Abnormal increase in Rad51 expression favors tumor progression by inhibiting the caspase-3-mediated apoptosis. In concert with the anti-apoptotic Bcl-2 family members, Rad51 overexpression results in diminished DNA damage. Elevated Rad51 may also interfere with other intracellular pathways, including p53, p21 and Bcl-2, which may cause improper repairing of the damaged DNA or further amplify the damaged sites in recombinant DNA strand [25]. Lastly, overexpression of Rad51 may also interfere with the G2 tetraploid checkpoint, thereby causing the formation of aneuploidy [26]

Rad51 expression has been considered an important indicator of tumor progression or remission in the multivariate analysis [8]. It was reported that Rad51 expression in invasive ductal breast carcinoma was higher than in normal breast tissue, and was significantly correlated with the pathological stage [16]In our study, although we did not note a significant correlation of Rad51 with CRC tumor stage, we found Rad51 expression was markedly higher in poorly differentiated carcinoma compared to the well differentiated carcinoma, supporting the observation that Rad51 is commonly associated with malignant histophenotypes. More significantly, we found Rad51 was higher in CRC patients with lymph node metastasis than those without, indicating that Rad51 overexpression may promote metastasis of CRC cells.

RETRACTED

Given the role of Rad51 in a variety of tumors, there was a growing interest in developing Rad51 inhibitors for the clinical use. Thus far, three compounds, B02, A03, and A10 have been identified by the high-throughput screenings [27]. Initial testing in a preclinical study showed Rad51 targeting overcame imatinib resistance in chronic myeloid leukemia [13]. A separate study with the mouse xenograft model has also showed the B02 compound was able to potentiate the anti-cancer effect of chemotherapeutic agents including doxorubicin, etoposide, topotecan, and cisplatin [28].

Collectively, our study is among the first to report the evidence of Rad51 overexpression in CRC with metastasis. Patients with lymph node metastasis generally have poor prognosis, and our data from the study population confirmed that Rad51 predicts poor prognosis in CRC. This view was further supported by the finding that CRC patients with Rad51 overexpression had significantly shorter survivals than those without. A similar study with a cohort of 383 non-small cell lung cancers also revealed that patients with strong Rad51 expression had significantly shorter survival than those with weak Rad51 expression [17]. Although significant further work is needed to understand the underlying mechanism, our current work suggests that Rad51 may serve as a valuable candidate for developing novel therapies in CRC.
